The article "Impaction Of Rehabilitations And Strengthening Programs before And after Anterior Cruciate Ligament Reconstruction In Return to the Fitness Level" was retracted in 2023. Reasons: unreliable results or conclusions; concerns about the data; concerns about the results or conclusions; concerns about the peer review.

# Impaction Of Rehabilitations And Strengthening Programs before And after Anterior Cruciate Ligament Reconstruction In Return to the Fitness Level

**DOI:** 10.1155/2022/7906341

**Published:** 2022-07-09

**Authors:** Abdulwahab Ahmed Alzahrani

**Affiliations:** Surgery Department, Faculty of Medicine, Albaha University, Pediatric Orthopedic & Deformities Fellow (WIEN), Consultant Orthopedic. Director of Orthopedic Resident Training Program, Albaha 65561, Saudi Arabia

## Abstract

**Objectives:**

Sports injuries are one of the most common orthopedic injuries particularly in young and active populations. Football is the most popular sport among Saudis, and thus, anterior cruciate ligament (ACL) injuries are common in clinics and emergency rooms in Saudi Arabia. The aim of this study was to evaluate the outcomes of patients six months after ACL reconstruction in both hospitals and gym-based rehabilitation services and its impaction on the patients to return to sports and preinjury fitness levels.

**Methods:**

This is a retrospective case series of patients who underwent arthroscopically assisted ACL reconstruction using a hamstring autograft at our center. Data were gathered from January 2020 to December 2020. Patients were given a questionnaire about their visits to the orthopedic clinic in the 6^th^ month after surgery.

**Results:**

Sixty patients with ACL reconstructions were studied. Noncontact sports were the leading cause of injuries (53.3%). The mean Lysholm score was 84.9 (SD 3.45) out of 100 after six months of follow-up, and the mean Tegner score was 4.77 (SD 1.06) out of 10 points. The Lysholm score was excellent (>90) among 5% (*n*= 3), good (84–90) among 60% (*n*= 36), and fair (65–83) among 35% (*n*= 21). As a result, we observed that the duration of postoperative rehabilitation has a significant relationship with the fitness level (*X*2= 18.711; *p*=0.001).

**Conclusion:**

The Lysholm knee scoring scale and the Tegner activity scale showed that arthroscopically assisted ACL reconstruction using hamstring autograft has a successful and functional outcome after which the patient returns to sports or regains the preinjury level of fitness level depends on the rehabilitation.The period and types of preoperative and postoperative rehabilitation have a direct impact on the return to fitness levels and normal daily life activities.

## 1. Introduction

Anterior cruciate ligament (ACL) injuries are common in clinics and emergency rooms. The ACL is the knee's primary stabilizer and prevents femur translation onto the tibia. In the United States, there are over 127,000 ACL reconstruction surgeries and 250,000 new ACL cases per year. [1] Discomfort while walking, inflammation, weakness, and signs of knee instability such as giving way and a reduction in athletic activities are all symptoms of ACL rupture [2].The gold standard surgical treatment is graft reconstruction followed by intensive rehabilitation [3]. A patient with ACL injury has a significant decrease in the activity, daily living, and low knee functional indicators, especially with a bilateral knee involvement [4]. Hamstring muscle tendon autograft has less complication rate in comparison to other autograft options. [5–7].

Preoperative and postoperative rehabilitation protocol exercise in the hospital and at the gym is crucial to returning to normal daily life activities. Physiotherapy is expected for at least two months with a minimum of four sessions per week. Restoring to full sport activities is contingent on completing a postoperative workout program, which can be completed six months after surgery [8]. The period of rehabilitation and the extent of the strengthening exercise program are strongly linked to a quick return to daily life activities and fitness levels [9]. The aim of this study was to identify and assess patients' functional outcomes six months after ACL reconstruction and their return to sports and daily life activities via both hospital- and gym-based rehabilitation, by using reliable and applicable international scoring tools. Two numerical rating questionnaires, which were introduced in 1985 by Tegner and Lysholm, were used to assess functional knee instability [10].

## 2. Materials and Methods

This was a retrospective case series of patients who underwent arthroscopically assisted ACL reconstruction using hamstring autografts at King Fahad Hospital in the Al-Baha region of Saudi Arabia.

This site is designated as a tertiary hospital by the Ministry of Health (MOH). Patients were treated and managed by one experienced arthroscopic surgeon. Hamstring autograft was used to treat all patients.

### 2.1. Procedures

All patients received the same preoperative instructions including prophylactic antibiotics and shaving 30 minutes prior to anesthesia. Spinal anesthesia was used in all patients, and the pivot test was used as the final diagnostic tool. Patients were placed in a supine position with a hanging leg in a leg holder; the tourniquet was applied at 250 mm Hg. Landmarks were placed using anteromedial and anterolateral portals.

### 2.2. Surgical Technique

Gracilis and semitendinosus tendons were harvested then sutured with sutures (Ethibond) using the Krackow technique. This followed the release of the bands attached to each tendon.

An incision was made for imaging, and a camera was inserted through the lateral port. The instrument was inserted through the medial port. The medial and lateral menisci, ACL, posterior cruciate ligament (PCL), and medial and lateral femoral condyles of the knee were inspected. The ACL traces at the insertion and origin sites were shaved away which spared some of the foot print at the tibial site for proprioception. 

Tibial tunneling was done at the middle of the ACL footprint. The tibial guide was inserted approximately 7 mm anterior to the PCL and 2–3 mm anterior to the tip of the medial spine. Reaming was done after insertion of a Kirschner wire (K-wire) through the tibial guide.

Femoral tunneling used an accessory anteromedial port with insertion of the femoral guidewire behind the footprint of the native ACL. The knee was then flexed more than 110°.

For graft passage, the suture loop was passed through the femoral tunnel followed by a crocodile pass of the suture along the tibial tunnel. The end button and an absorbable interference screw was used along with a stapler to secure the graft while tensioning it in an extended knee position. Finally, the patient was put in a knee stabilizer.

From January 2018 to December 2019, data were collected from 68 patients who met the inclusion criteria, except for eight patients who were unable to participate in the research study. The patients were all males between 19 and less than 45 years old with no comorbidities and a body mass index (BMI) in-between 19 and 30. All subjects had an isolated ACL tear and could perform postoperative recovery exercises. Sixty patients were involved in this study. Questionnaires were distributed to the patients six months after their orthopedic surgery. All subjects gave informed verbal consent before participating in the questionnaires.

The Lysholm score and the Tegner scales were used to assess patient outcomes. The Lysholm Scale is a reliable scoring system that includes the following eight elements: discomfort, swelling, limping, squatting, locking, instability, stair climbing, and the need for help [1]. The return to daily life activities and the normal level of fitness were assessed using direct questions.

### 2.3. Statistical Analysis

When applicable, the data were presented in the form of numbers, percentages, means, and standard deviations. The independent *t*-test and one-way ANOVA were used to compare the Lysholm and Tegner scores to patients' diagnostic criteria.

Fischer's exact test was used to investigate the relationship among restoring the fitness level, recovery extent, and recovery period. In all statistical studies, a *P* value of 0.05 was considered significant. All statistical analyses for this project were performed using Statistical Packages for Social Sciences (SPSS) version 21 (IBM Corporation in Armonk, New York).

## 3. Results

We analyzed sixty patients who underwent ACL reconstruction. The clinical characteristics of the patients with ACL injury are listed in Table 1. The most common cause of injury was noncontact sports (36.7%) followed by contact sports (36.7%). More than half of those surveyed (51.7%) injured their dominant leg.

The main concern of 71.7% of the patients was instability. Furthermore, 51.7% had a gap of more than a year between the injury and the surgery. The most common types of rehabilitation (43.3%) were regular hospital rehab and gym rehab, and the most common rehabilitation period was less than a month (36.7%).

Likewise, one-third of the patients expressed an interest in resuming their previous level of fitness. The mean Lysholm and Tegner scores were 84.9 and 4.77, respectively, with an average of 8.98 weeks for returning to normal daily activities.

Figure 1 presents the Lysholm score categories: 60% of the patients (*N*= 36) had a good score(84–90), 35% of the patients (*N*= 21) had a fair score (65–83), and only 5% of the patients (*N*= 3) had an excellent score (>90).

When the Lysholm and Tegner scores were compared to the clinical characteristics of the patients, we found that those who did not participate in a recovery program had substantially lower Lysholm (*F*= 7.895; *p* < 0.001) and Tegner (*F*= 7.233; *p* < 0.001) scores. Similarly, there was a substantial difference in Lysholm (*F*= 4.749; *p* < 0.001) and Tegner scores (*F*= 4.640; *p*=0.001) with the period of postoperative recovery.

Furthermore, those who returned to their previous fitness levels had substantially higher Lysholm (*T*= 6.537; *p* < 0.001) and Tegner (*T*= 7.317; *p* < 0.001) scores. When then compared both Lysholm and Tegner ratings with other clinical features of the patients such as the mode of injury, dominant leg, and time between the injury and the surgery. There was no substantial difference (all *p* > 0.05).  Table 2 shows the statistical difference between Lysholm and Tegner scores in relation to the clinical characteristics of patients with ACL injury (*n*= 60).

Figure 2 shows the correlation between Lysholm and Tegner scores. Correlation between Lysholm and Tegner scores was positively highly and statistically significant (*r*= 0.827; *p* < 0.001), and the Lysholm knee score and the Tegner activity scale demonstrated acceptable psychometric performances as outcome measures for patients with knee injury.

Figure 3 shows the correlation between the Lysholm score and returning to normal daily activities time in weeks. There was a highly but inverse correlation between the Lysholm score and returning to normal daily activities time in weeks (*r*= -0.694; *p* < 0.001).

Figure 4 shows the correlation between the Tegner score and the time needed to return to normal daily activities in weeks. There was a negative highly significant correlation between the Tegner score and that time interval (*r*= -0.713; *p* < 0.001).

We then compared the period of postoperative rehabilitation to the return to the fitness level: the duration of postoperative rehabilitation had a substantial impact (*X*2= 18.711; *p*= 0.001), but the form of rehabilitation did not have the similar impact (*X*^2^= 2.724; *p*= 0.005).  Table 3 shows the relationship between returning to the fitness level and the type of rehabilitation including rehabilitation duration (*n*= 60).

## 4. Discussion

The results revealed that the patients' functional outcomes were generally good. According to the Lysholm knee-scoring scales, the mean score was 84.9 (3.45) out of 100 with 60% of the patients having good results (Lysholm score 84–90); 35% had fair results (Lysholm score 65–83), and the remaining 5% had excellent results (>90). The grading system was obtained from the study of Misou et al. [11] A Pakistani study found that more patients had excellent functional outcomes as calculated by the Lysholm knee scoring scale after ACL reconstruction [12,13]. In India, [14] a case series of 25 patients who underwent ACL reconstruction for a year and were operated on by a single surgeon found that the mean preoperative Lysholm score was 58.8 (fair 56%; bad 44%). This increased to 91.2 after surgery (excellent 72%; good 24%). This was also higher than our findings. On the other hand, our findings are consistent with Devgan et al. [15] and Bangert and colleagues [16].(The average postoperative Lysholm score was 86 in both studies). The Tegner activity scale was another significant indicator for determining the patients' functional status. After six months of follow-up, the patients' mean Tegner score was 4.77 (1.06) out of 10 points. The Tegner score used in our study was consistently within the recorded range as defined by the literature [13, 15].

Patients who participated in both a hospital and gym rehab program for more than two months had a higher functional ability than those who participated in either a hospital rehab or a gym rehab program only. We also discovered that patients who regained their health had a higher functional status than those who did not. We also observed that the association between Lysholm and Tegner scores was significantly higher (*p*= 0.001), thus implying that the Tegner score increased with the Lysholm score.

However, the association between Lysholm and Tegner scores in relation to time spent returning to normal daily life activities were highly inversely correlated (*p*= 0.001), implying that an increase in Tegner performance corresponds to a decrease in weeks spent returning to normal daily life activities. Furthermore, we found that the length of postoperative rehabilitation has a significant impact on returning to the fitness level (*p*= 0.001).

To the best of our knowledge, only a few articles have examined the impact of the Lysholm and Tegner scores on postsurgery patient characteristics.

These findings are a valuable addition to this study discipline's ongoing research. More than half of the subjects (51.7%) had a duration of more than one year between the incident and the procedure, and these may be attributed to the fact that 53.3% of the cases involved noncontact sports. Shaikh et al. [12]stated that most cases had surgery within six months of the date of injury, which is shorter than our study. This is most likely because most cases recorded were as a result of a car accident that necessitated abrupt intervention or surgery.

According to Chodavarapu and associates [14], the most common presurgical concern was instability. This supports the findings of Devgan and colleagues [15] who found that patients experienced persistent knee pain and instability before arthroscopic assisted ACL reconstruction.

## 5. Conclusion

The Lysholm knee scoring scale and the Tegner activity scale show that arthroscopically assisted ACL reconstruction with a hamstring autograft has a successful functional outcome after rehabilitation. More than two months of regular postoperative recovery in both hospital and gym rehabilitation programs are a significant step in regaining fitness. The duration of postoperative recovery has a significant impact on resuming regular daily life activities and fitness levels.

Therefore, we first strongly emphasize preventing ACL injury by strength training of the quadriceps and hamstrings along with muscles and ligaments of the feet and ankles.

These prevention steps can prevent the pivoting or twisting that leads to ACL tears. We also recommend stretching and warming up these ligaments and muscles prior to any intense activities.

We further recommend educating patients with torn ACLs about the importance of having good strengthening and training programs (swimming and stationary bicycle exercises) before surgery. Surgery should be followed with extensive rehabilitation therapy at a hospital under supervision of a professional therapist after ACL reconstruction surgery. Finally, we recommend an exercise program that strengthens the whole lower limb muscles and ligaments, especially quadriceps, hamstring, ankles, and feet.

## Figures and Tables

**Figure 1:** Postoperative Lysholm score.

**Figure 2:** Correlation (Pearson-r) between Lysholm and Tegner scores.

**Figure 3:** Correlation (Pearson's (R) between the Lysholm score and the time needed to return to normal daily activities (weeks).

**Figure 4:** Correlation (Pearson's (R) between the Tegner score and the time needed to return to normal daily activities (weeks).

**Table 1:** Clinical characteristics of patients with an ACL injury (*n*= 60).

Variables	N (%)
Mode of injury	
(i) Road traffic accident (RTA)	01 (01.7%)
(ii) Falling	05 (08.3%)
(iii) Contact sport	22 (36.7%)
(iv) Noncontact sport	32 (53.3%)

Dominant leg	
(i) Right	31 (51.7%)
(ii) Left	29 (48.3%)

Chief complaint	
(i) Instability	43 (71.7%)
(ii) Locking	04 (06.7%)
(Iii) Both	13 (21.7%)

Duration between the injury and the surgery	
(i) < 6 months	08 (13.3%)
(ii) > 6 months and <1 year	21 (35.0%)
(iii) > 1 year	31 (51.7%)

Types of rehabilitation	
(i) Standard hospital rehab program	20 (33.3%)
(ii) Gym rehab	11 (18.3%)
(iii) Both	26 (43.3%)
(iv) None	03 (05.0%)

The duration of post-operative rehabilitation	
(i) Less than one month at the hospital	13 (21.7%)
(ii) More than two months at the hospital	07 (11.7%)
(iii) Less than one month at a gym	02 (03.3%)
(iv) More than two months at a gym	09 (15.0%)
(v) Less than one month in both	04 (06.7%)
(vi) More than two months in both	22 (36.7%)
(vii) None	03 (05.0%)

Returning to the fitness level	
(i) Yes	20 (33.3%)
(ii) No	40 (66.7%)

	Mean ± SD
Lysholm scoring scale	84.9 ± 3.45
Tegner score	4.77 ± 1.06
Returning to normal daily activities in weeks	8.98 ± 1.35

**Table 2:** Statistical difference between Lysholm and Tegner scores in relation to the clinical characteristics of patients with ACL injury (*n*= 60).

Factor	Lysholm score	F/*T*-test;	Tegner score	F/*T*-test;
	Mean ± SD	*P* value	Mean ± SD	*P* value
Mode of injury^a^				
(i) Road traffic accident (RTA)/Falling	84.7 ± 4.93	*F*= 0.815; 0.448	4.67 ± 1.37	*F*= 1.214; 0.305
(ii) Contact sport	85.6 ± 3.54		5.05 ± 1.13	
(iii) Noncontact sport	84.4 ± 3.09		4.59 ± 0.95	

Dominant leg^b^				
(i) Right	84.9 ± 3.83	*T*= 0.048; 0.962	4.65 ± 1.11	*T*= -0.914; 0.365
(ii) Left	84.8 ± 3.06		4.89 ± 1.01	
Chief complaint^a^				
(i) Instability	85.2 ± 3.27	*F*= 1.804; 0.174	4.84 ± 0.92	*F*= 1.363; 0.264
(ii) Locking	86.0 ± 3.37		5.25 ± 1.50	
(iii) Both	83.3 ± 3.84		4.38 ± 1.33	

Duration between the injury and the surgery^a^				
(i) < 6 months	83.4 ± 3.29	*F*= 1.569; 0.217	4.38 ± 0.92	*F*= 1.794; 0.176
(ii) < 1 year	85.8 ± 3.21		5.09 ± 1.09	
(iii) > 1 year	84.6 ± 3.57		4.65 ± 1.05	

Types of rehabilitation^a^				
(i) Hospital rehab program	83.8 ± 2.95	*F*= 7.895; **<0.001**^*∗∗*^	4.40 ± 0.94	*F*= 7.233; **<0.001**^*∗∗*^
(ii) Gym rehab	84.5 ± 2.91		4.73 ± 0.90	
(iii) Both	86.5 ± 3.11		5.27 ± 0.96	
(iv) None	78.7 ± 0.58		3.00 ± 0.00	

Duration of postoperative rehabilitation^a^					
(i) Less than one (1) month at the hospital	82.8 ± 2.79	*F*= 4.749; **0.001**^*∗∗*^	4.08 ± 0.86	*F*= 4.640; **0.001**^*∗∗*^
(ii) More than two months at the hospital	85.6 ± 2.51		5.00 ± 0.82	
(iii) Less than one month at a gym	83.5 ± 3.54		4.50 ± 0.71	
(iv) More than two months at a gym	84.8 ± 2.95		4.78 ± 0.97	
(v) Less than one month in both	86.3 ± 4.03		5.00 ± 0.82	
(vi) More than two months in both	86.5 ± 3.04		5.32 ± 0.99	
(vii) None	78.7 ± 0.58		3.00 ± 0.00	

Returning to the previous fitness level^b^				
(i) Yes	88.0 ± 2.47	*T*= 6.537; **<0.001**^*∗∗*^	5.80 ± 0.83	*T* = 7.317; **<0.001**^*∗∗*^
(ii) No	83.3 ± 2.72		4.25 ± 0.75	

Most authors use the terms statistically significant (P 0.05) and statistically highly significant (P 0.001). ( Less one in a thousand chance of being wrong). The outcome is regarded as extremely significant.

**Table 3:** Relationship between returning to the fitness level and the type of rehabilitation including rehabilitation duration (*n*= 60).

Factor	Returning to fitness level			*P* value^§^
	Yes N (%) ^(n=^^20)^	No N (%) ^(n=^^40)^	X^2^	
Type of rehabilitation				
(i) Standard hospital rehab program	06 (30.0%)	14 (35.0%)	2.724	0.552
(ii) Gym rehab	03 (15.0%)	08 (20.0%)		
(iii) Both	11 (55.0%)	15 (37.5%)		
(iv) None	0	03 (07.5%)		

The duration of postoperative rehabilitation				
(i) Less than one month at the hospital	0	13 (32.5%)	18.711	**0.001** ^*∗∗*^
(ii) More than two months at the hospital	06 (30.0%)	01 (02.5%)		
(iii) Less than one month at a gym	0	02 (05.0%)		
(iv) More than two months at a gym	03 (15.0%)	06 (15.0%)		
(v) Less than one month in both	02 (10.0%)	02 (05.0%)		
(vi) More than two months in both	09 (45.0%)	13 (32.5%)		
(vii) None	0	03 (07.5%)		

The result is considered highly significant if the P value is 0.001 or less.

## Data Availability

The datasets are available from the corresponding author either collected or analyzed during the current study on reasonable request and upon IRB approval.
